The article "Impact of Adjacent Facet Joint Osteoarthritis on Adjacent Segment Degeneration after Short-Segment Lateral Lumbar Interbody Fusion for Indirect Decompression: Minimum 5-Year Follow-Up" was published in 2022. Journal: Biomed Res Int.

# Impact of Adjacent Facet Joint Osteoarthritis on Adjacent Segment Degeneration after Short-Segment Lateral Lumbar Interbody Fusion for Indirect Decompression: Minimum 5-Year Follow-Up

**DOI:** 10.1155/2022/3407681

**Published:** 2022-08-22

**Authors:** Jun Ouchida, Hiroaki Nakashima, Tokumi Kanemura, Kotaro Satake, Kenyu Ito, Mikito Tsushima, Kei Ando, Masaaki Machino, Sadayuki Ito, Naoki Segi, Yoshinori Morita, Yukihito Ode, Shiro Imagama

**Affiliations:** ^1^Department of Orthopaedics, Nagoya University Graduate School of Medicine, Nagoya, Japan; ^2^Department of Orthopedic Surgery, Konan Kosei Hospital, Konan, Japan

## Abstract

**Purpose:**

Lumbar fusion combined with lateral lumbar interbody fusion (LLIF) and percutaneous pedicle screws (PPS) is a widely used, minimally invasive surgical treatment, but studies on incidence and risk factors for subsequent adjacent segment degeneration (ASD) are limited. This study was aimed at investigating midterm incidence and reoperation rate of ASD after indirect decompression (IDD) with LLIF and PPS and at clarifying the impact of preexisting adjacent facet osteoarthritis on development of ASD after IDD.

**Methods:**

Forty-one patients who underwent short-segment (1- or 2-level) lumbar fusion with LLIF and PPS with a minimum 5-year follow-up were analyzed. Cephalad adjacent facet osteoarthritis was classified as 1 (normal) to 4 (severe) by an established classification system on preoperative CT. ASD was diagnosed with plain radiographs taken preoperatively and up to 5 years postoperatively, and preoperative degree of facet osteoarthritis was compared between the ASD+ group and ASD- group (control). We also divided patients into two groups according to severity of facet degeneration, mild (grades 1-2) group and severe (grades 3-4) group, and investigated ASD-free survival of the groups by the Kaplan-Meier method.

**Results:**

The incidence of ASD at 5 years postoperatively was 34.1%, and the reoperation rate for ASD was 4.9%. The degree of preexisting facet joint osteoarthritis was significantly different between the ASD+ and ASD- groups (grade 1/2/3/4: 0/29/64/7% and 29/62/29/10%, *P* = 0.008). Kaplan-Meier analysis showed the severe group to have significantly lower ASD-free survival than the mild group (*P* = 0.017) at 5 years postoperatively.

**Conclusion:**

Comparative analysis of the ASD+ versus ASD- group showed preexisting facet joint osteoarthritis to be a risk factor for ASD progression after IDD. Additional longitudinal studies with long-term follow-up are needed to understand the causal relationship between facet joint degeneration and progression of adjacent segment deterioration following IDD.

The article "Impact of Adjacent Facet Joint Osteoarthritis on Adjacent Segment Degeneration after Short-Segment Lateral Lumbar Interbody Fusion for Indirect Decompression: Minimum 5-Year Follow-Up" was published in 2022. Journal: Biomed Res Int.

## 1. Introduction

Lumbar spinal fusion is the gold standard for surgical treatment of spinal degenerative diseases with instability, with a number of studies reporting favorable surgical outcomes [1–3]. Fixation surgery of the mobile lumbar spine alters the forces applied to adjacent mobile segments, resulting in accelerated degeneration of the adjacent spinal level, and has been reported as adjacent segment degeneration (ASD). Risk factors for the development of ASD are multifactorial, including preexisting facet degeneration, iatrogenic damage of posterior connective components due to surgery, and local lumbar and spinopelvic sagittal alignment [4–9].

In contrast, lumbar fusion using a lateral lumbar interbody fusion (LLIF) cage allows for indirect nerve decompression via the ligamentotaxis principle by restoring the intervertebral height, stabilizing the spine, and preserving the anterior longitudinal ligament, for which favorable results have been reported. [10, 11] Indirect decompression (IDD) using LLIF in combination with percutaneous pedicle screw (PPS) fixation has advantages in preserving posterior connective components, reducing intraoperative complications such as nerve injury and bleeding, and preventing adjacent facet joint violation by posterior implantation when intraoperative computed tomography (CT) navigation is used for screw insertion [2, 12]. We considered that the combination of restoration of the alignment of the degenerated intervertebral space by using a LLIF cage and PPS insertion technique with intraoperative CT navigation to preserve the superior adjacent facet joint would reduce the incidence of ASD and reoperation rate after lumbar fusion surgery. However, to our knowledge, there are few reports of postoperative ASD after 5indirect decompression surgery. Because of the paucity of information on this subject [13, 14], it is important to better understand the mechanism of development of ASD by investigating the incidence of postoperative ASD and the risk factors described above that are involved in its development following the use of this minimally invasive technique. Therefore, the purpose of this retrospective cohort study was to investigate the midterm incidence of cephalad ASD and reoperation rates after IDD surgery and to clarify the association of lumbar sagittal alignment and adjacent facet degeneration with the development of ASD after IDD by comparing an ASD+ group with an ASD- group. In this study, we defined the ASD+ group as patients radiographically having ASD and the ASD- group as those without ASD until the 5-year postoperative follow-up at which time clinical and radiographical outcomes were compared.

The article "Impact of Adjacent Facet Joint Osteoarthritis on Adjacent Segment Degeneration after Short-Segment Lateral Lumbar Interbody Fusion for Indirect Decompression: Minimum 5-Year Follow-Up" was published in 2022. Journal: Biomed Res Int.

## 2. Materials and Methods

### 2.1. Subjects

We retrospectively included 109 consecutive patients who underwent LLIF with PPS at a single institution between May 2013 and June 2016. The subjects were patients with more than 5 years of follow-up who underwent short-segment lumbar fixation between 1 or 2 vertebral levels for spinal degenerative diseases with spondylolisthesis and instability. To standardize the pathological baseline involving the adjacent facet joints of the patients in the analysis, patients with trauma, syndromic spine, spinal deformity, surgery for secondary pseudoarthrosis or ASD after lumbar fusion, or more than three levels of fusion were not included in this study. Patients with severe psychiatric disorders or adverse events that did not necessitate postoperative clinical and radiographical assessment were also excluded from our analysis. In all cases, anterior fixation with a LLIF cage was performed via a transpsoas approach, followed by posterior fixation using a PPS method aided by O-arm navigation (Medtronic Sofamor Danek, Inc., Memphis, TN). The LLIF and PPS surgical procedures were performed on the same day.  Figure 1 shows the flowchart of patient allocation in this study. This study was approved by the Institutional Review Board of Konan Kosei Hospital, Konan, Japan, and written informed consent was waived because of the retrospective design of the study.

### 2.2. Assessment of Adjacent Segment Degeneration

On the basis of previous reports [5, 15], we defined ASD+ as the proximal adjacent level containing any of the following three conditions on a lateral radiograph: (1) postoperative vertebral slippage of ≥3 mm, (2) narrowing of the intervertebral space of ≥3 mm, or (3) postoperative intervertebral opening of ≥5%. Residual neurological symptoms as noted in the medical records at follow-up and reoperation rates at 5 years postoperatively were also investigated.

Clinical outcomes of reoperation rate, Japanese Orthopaedic Association (JOA) score, and residual neurological symptoms and radiographical outcomes of bony fusion on plain radiograph and deterioration of ASD and changes of dural sac cross-sectional area on magnetic resonance imaging (MRI) were measured and evaluated. Bony fusion was defined as the presence of obvious bony continence in the anterior or posterior column of the fixed levels on a lateral radiograph. Disc degeneration was assessed using the Pfirrmann grading system [16], and dural sac cross-sectional area was measured manually using picture archiving and communication systems (Hope Dr Able-GX, Fujitsu Co., Tokyo, Japan).

### 2.3. Factors Affecting ASD Progression

To investigate the factors affecting ASD progression, we compared the patient profiles and perioperative radiographical parameters between the ASD+ and ASD- groups. The comparative variables between the two groups were age, sex, number of fixation levels, degree of cephalad adjacent facet joint osteoarthritis on preoperative CT, degree of adjacent disc degeneration on preoperative MRI, facet violation by the PPS (screw invasion into the cortex of the facet joint) on postoperative CT, pelvic incidence (PI), pelvic tilt (PT), sacral slope (SS), lumbar lordosis (LL), PI-LL mismatch, acquisition of local lordosis, and acquisition of intervertebral height for sagittal alignment on the 2-week postoperative radiograph. The intervertebral height was defined as the average measurement of intervertebral distance at the anterior and posterior edges on a plain lateral radiograph. Local lordosis acquisition and local intervertebral height restoration were calculated by the difference in values of the preoperative and postoperative radiographical parameters for each fixed level. In cases with multilevel fixation, the average of each value was used for analysis. The severity of osteoarthritis of the adjacent facet joint was classified from grades 1 (normal) to 4 (severe) on the preoperative axial CT images, referring to the classification of Kalichman et al. [17]. Representative images of each grade are shown in Figure 2. We used these grades to classify the degeneration of the cephalad adjacent facet joint and further divided the patients into the mild (grades 1-2) group and severe (grades 3-4) group to analyze the impact of the severity of preexisting facet joint osteoarthritis on the ASD-free survival rate at 5 years after surgery.

The article "Impact of Adjacent Facet Joint Osteoarthritis on Adjacent Segment Degeneration after Short-Segment Lateral Lumbar Interbody Fusion for Indirect Decompression: Minimum 5-Year Follow-Up" was published in 2022. Journal: Biomed Res Int.

### 2.4. Statistical Analysis

All values are expressed as means ± standard deviation. The paired *t*-test was used to compare continuous variables before and after the surgery, and the Mann-Whitney *U* test was used to determine significant differences between the two groups for continuous variables and ordered variables. Fisher's exact test was used for univariate analysis including categorical variables. The incidence of ASD was analyzed using Kaplan-Meier survival analysis. Statistical significance was set at *P* < 0.05. IBM SPSS Statistics version 23.0 software (IBM Corp., Armonk, NY) was used for statistical analyses.

## 3. Results

Of the 109 patients who underwent short-segment LLIF and PPS, 41 patients were included in the analysis. Patient demographic data and surgical outcomes are shown in Table 1. The mean age of the 18 males and 23 females was 70.0 ± 7.2 years. The preoperative diagnosis was degenerative spondylolisthesis (grade 1, 31 cases; grade 2, 2 cases) in 33 cases and spinal canal stenosis in 8 cases. The levels of fixation were L3/4 and L4/5 in 7 and 24 cases, respectively, and L3-5 for two levels in 10 cases. Regarding clinical outcome, the JOA score was 14.8 ± 4.3 points preoperatively and 25.8 ± 2.5 points postoperatively (*P* < 0.001 vs. preoperatively). The respective pre- and postoperative radiographical parameters on plain radiographs were 41.2 ± 12.4 and 44.1 ± 13.4 degrees (*P* = 0.007) for LL, 9.1 ± 11.8 and 6.2 ± 12.0 degrees (*P* = 0.007) for PI-LL mismatch, 6.9 ± 7.2 and 13.1 ± 5.2 degrees (*P* < 0.001) for local lordosis, and 8.6 ± 4.2 and 13.8 ± 4.7 mm (*P* < 0.001) for intervertebral height.

The article "Impact of Adjacent Facet Joint Osteoarthritis on Adjacent Segment Degeneration after Short-Segment Lateral Lumbar Interbody Fusion for Indirect Decompression: Minimum 5-Year Follow-Up" was published in 2022. Journal: Biomed Res Int.

In the preoperative evaluation of the adjacent level, the degree of facet joint osteoarthritis was grade 1 in 6 cases (14.6%), grade 2 in 17 cases (41.5%), grade 3 in 15 cases (36.6%), and grade 4 in 3 cases (3.0%) according to the Kalichman classification, and the degree of adjacent disc degeneration was grade 1 in 0 cases, grade 2 in 1 case, grade 3 in 7 cases, grade 4 in 24 cases, and grade 5 in 9 cases according to the Pfirrmann grading system. The dural sac cross-sectional areas on pre- and postoperative MRI were 147.3 ± 36.4 mm^2^ and 140.3 ± 37.6 mm^2^, respectively (*P* = 0.005). Cephalad adjacent facet joint violation by PPS was observed in 2 patients.

At the end of 5 years of follow-up, 14 patients (34.1%) were diagnosed as having ASD according to the criteria. Two patients (4.9%) in the ASD+ group underwent reoperation for ASD, with both undergoing extension of fixation for cephalad adjacent segment deformity. One patient in the ASD- group underwent additional fixation for caudal foraminal disc herniation. There were no significant differences in the reoperation rate for ASD (*P* = 0.111), change in the JOA score (−2.3 ± 3.4 vs. −1.1 ± 3.2 points, *P* = 0.266), residual neurological symptoms (28.6 vs. 22.2%, *P* = 0.712), and bony fusion rate (92.9 vs. 85.9%, *P* = 0.645) on radiographs between the ASD+ and ASD- groups at the final follow-up. There were, however, significant differences in the deterioration of disc degeneration (85.7 vs. 22.2, *P* < 0.001) and percent change of the dural sac cross-sectional area (−28.1 ± 25.3 vs. −10.4 ± 22.4%, *P* = 0.027) between the two groups (Table 2).

Univariate analysis of ASD risk factors showed no significant differences between the ASD+ group and ASD- group in age (71.1 ± 7.6 vs. 69.4 ± 7.0 years, *P* = 0.494), sex (50.0 vs. 59.3%, *P* = 0.742), number of fixation levels (2 levels, 42.9 vs. 14.8%, *P* = 0.064), facet joint violation by PPS (14.3 vs. 0%, *P* = 0.111), radiographical parameters at 2 weeks postoperatively, and preoperative adjacent disc degeneration (grade 1/2/3/4/5: 0/1/6/7/0 vs. 0/1/12/12/2, *P* = 0.566). However, there was a significant difference in the degree of preexisting facet joint osteoarthritis (grade 1/2/3/4: 0/4/9/1 vs. 6/13/6/2, *P* = 0.008) (Table 3).

The article "Impact of Adjacent Facet Joint Osteoarthritis on Adjacent Segment Degeneration after Short-Segment Lateral Lumbar Interbody Fusion for Indirect Decompression: Minimum 5-Year Follow-Up" was published in 2022. Journal: Biomed Res Int.

Kaplan-Meier analysis of ASD-free survival for preexisting facet joint osteoarthritis showed that at 5 years postoperatively, the grade 3-4 group had significantly more ASD than the grade 1-2 group (*P* = 0.017) (Figure 3).

### 3.1. Illustrative Case

An illustrative case of ASD is shown in Figure 4. A 61-year-old woman underwent lumbar fusion of L4/5 with LLIF and PPS for grade 1 spondylolisthesis. A preoperative CT axial view showed overall narrowing of the facet joint of the L3/4 and a subchondral cyst (grade 3). The JOA score improved from 14 points preoperatively to 28 points postoperatively. At 2 years postoperatively, posterior slippage of the L3 vertebra and decrease in L3/4 disc space height were found on a plain lateral radiograph. MRI showed a decrease in the dural sac cross-sectional area from 178 mm^2^ at 2 weeks after surgery to 114 mm^2^ (-36% change) at the last follow-up and thickening of connective tissue and ligaments around the facets and posterior protrusion of the L3/4 disc.

## 4. Discussion

In this study, radiographical ASD was found to be associated with degenerative changes in the intervertebral disc at the adjacent level and a decrease in the dural sac cross-sectional area on MRI. In a univariate analysis of the ASD+ group and ASD- group, the degree of preoperative facet joint osteoarthritis, rather than sagittal alignment (LL, PI, PT, etc.) or local lordosis of the fixation level, was shown to be a significant risk factor for developing ASD after IDD surgery. We hypothesized that sagittal alignment and local lordosis formation on radiographs would also be associated with the development of ASD even in LLIF surgery combined with PPS as in conventional lumbar fusion, but no significant difference was found in this study. Interestingly, the present results did not show an association of ASD with preexisting disc degeneration, indicating that the degree of preoperative facet joint osteoarthritis is independently significant, and preoperative CT evaluation of the adjacent facet joints is recommended to estimate the risk of postoperative reoperation or to determine the range of fusion levels before an initial surgery.

Radiographical evidence of degeneration in an adjacent segment of the fixed levels indicates the potential for progression to a symptomatic condition and often results in reoperation. Previous studies of lumbar fusion with comparable postoperative follow-up periods to that of the present study have reported an incidence of radiographical ASD of 31–49%, with reoperation rates of 12–17% [7, 15, 18–20]. The incidence of ASD of 34.1% in the present study was comparable, whereas the rate of reoperation of 4.9% was lower than that of past reports. On the basis of the previously reported results of lumbar fusion surgery with LLIF [2, 21], we hypothesized that the acquisition of sufficient local lordosis and LL by LLIF surgery would be advantageous in reducing postoperative ASD occurrence, even in short-segment lumbar fusion [22, 23]. Lee et al. [24] reported in a comparative study of short-segment lumbar fusion including LLIF and posterior lumbar interbody fusion (PLIF) that LLIF was superior to PLIF in terms of intervertebral height adjustment and the incidence of ASD at 41.7% and 64.5%, respectively. Bae et al. [25] reported an ASD incidence rate of 10.6% in a study of more than 3 years of follow-up after lumbar fusion with LLIF and PPS and described segmental lordosis and LL as risk factors for the development of ASD. Although both of these reports show the incidence of ASD after lumbar fusion with LLIF, the present study is the first, to our knowledge, to show 5-year follow-up results. However, this study did not focus on the advantage of LLIF compared to PLIF with regard to the acquisition of alignment. The potential benefit of LLIF over PLIF and transforaminal lumbar interbody fusion in reducing the incidence of ASD remains controversial [14], and longer-term comparative studies are needed to standardize the criteria for ASD diagnosis and baseline patient profiles, such as the severity of spondylolisthesis.

The article "Impact of Adjacent Facet Joint Osteoarthritis on Adjacent Segment Degeneration after Short-Segment Lateral Lumbar Interbody Fusion for Indirect Decompression: Minimum 5-Year Follow-Up" was published in 2022. Journal: Biomed Res Int.

A number of studies have been conducted on risk factors for ASD, and instrumentation, fusion length, sagittal malalignment, and posterior connective component damage due to surgery have been reported as independent factors in the development of ASD [4, 6–9]. An occurrence of ASD is the result of a multifactorial pathology, although sagittal alignment and reduction of posterior tissue damage due to surgery have been proposed as variables that can be resolved by developing an appropriate surgical strategy [6, 21, 26, 27]. A comparative analysis of the ASD+ and ASD- groups showed no significant differences in the postoperative acquisition of local lordosis or in intervertebral height; however, preexisting adjacent facet joint osteoarthritis was found to be a risk factor for the development of postoperative ASD. Furthermore, the 5-year postoperative ASD-free survival curve showed that the group with more severe facet joint osteoarthritis had fewer ASD-free cases than the milder group. Lee et al. [8] reported the development of ASD requiring reoperation in 2.6% of more than 1000 patients who underwent lumbar fusion and discussed that preoperative preexisting facet joint degeneration was a risk factor for the development of ASD postoperatively, and Yoshiiwa et al. [28] reported that facet joint degeneration was associated with thickening of the ligamentum flavum in a study analyzing CT and MRI findings in patients with neurological symptoms. The presence and progression of facet degeneration are thought to be strongly related to the pathogenesis of nerve compression, such as disc protrusion and thickening of the ligamentum flavum, and the evaluation and preservation of adjacent facet joint degeneration are essential for the estimation and prevention of symptomatic ASD progression even after lumbar stabilization surgery with LLIF and PPS.

The article "Impact of Adjacent Facet Joint Osteoarthritis on Adjacent Segment Degeneration after Short-Segment Lateral Lumbar Interbody Fusion for Indirect Decompression: Minimum 5-Year Follow-Up" was published in 2022. Journal: Biomed Res Int.

There are several limitations that should be considered in our study. First, a 5-year period of postoperative follow-up may be insufficient for discussing ASD after lumbar fusion. Nakashima et al. [5] reported that 80% of revision surgeries for ASD were performed more than 5 years after the initial surgery in a study that followed patients for more than 10 years after lumbar fusion, and several studies reported a constant incidence of ASD up to 10 years after surgery [15, 20]. Second, this study only included the cephalad ASD of short-segment IDD, which may not cover the comprehensive risk factors of ASD after lumbar fusion. One patient in this study group also underwent revision surgery of the caudal level, and the contribution of the lower lumbar lesion to clinical outcomes could not be clarified in this analysis. Third, the number of cases in this study is small, and thus, future multicenter studies that include a larger number of cases will be needed to reduce potential bias in clinical outcomes caused by specific surgeons or single centers. Even with these limitations, we believe that the results of this study, which focused on cephalad ASD after IDD under intraoperative CT navigation guidance, will help the surgeon to choose a surgical strategy that preserves the cephalad adjacent facet joint and make an appropriate preoperative prognostic assessment of ASD.

## 5. Conclusions

Among all cases, the incidence of cephalad ASD at 5 years after lumbar fusion for IDD combined with LLIF and PPS was 34.1%, and the reoperation rate for ASD was 4.9%. Comparative analysis between the ASD+ and ASD- groups found preexisting adjacent facet joint osteoarthritis to be a risk factor for ASD progression, with no significant differences in sagittal parameters or pre- and postoperative local alignment. Additionally, longitudinal studies with long-term follow-up will be needed to understand the causal relationship between facet joint degeneration and progression of adjacent segment deterioration subsequent to IDD.

The article "Impact of Adjacent Facet Joint Osteoarthritis on Adjacent Segment Degeneration after Short-Segment Lateral Lumbar Interbody Fusion for Indirect Decompression: Minimum 5-Year Follow-Up" was published in 2022. Journal: Biomed Res Int.

## Figures and Tables

**Figure 1:** Flow diagram with number of patients included. Of 109 patients treated with LLIF and PPS, 41 patients who underwent LLIF+PPS for lumbar degenerative disease and were followed up for at least 5 years were analyzed. Fourteen patients were diagnosed as having ASD (ASD+ group), and 27 were diagnosed as not having ASD (ASD- group (control)). LLIF: lateral lumbar interbody fusion; PPS: percutaneous pedicle screw; ASD: adjacent segment degeneration.

**Figure 2:** Facet joint osteoarthritis grade. (a) Grade 1 (normal): facet joint space is preserved, and there is no osteosclerosis or facet hypertrophy. (b) Grade 2 (mild): facet joints with mild osteoarthritis. Joint space narrowing, sclerosis, and facet hypertrophy are present. (c) Grade 3 (moderate): facet joints with moderate osteoarthritis. Osteophytes (white arrow), subchondral cysts (black arrow), and vacuum phenomenon are present. (d) Grade 4 (severe): facet joints with severe arthritis. Overall narrowing of the joint space, large osteophytes (white arrow), facet hypertrophy, subchondral cysts (black arrow), and vacuum phenomenon (gray arrow) are present.

**Figure 3:** Kaplan-Meier survival curve of adjacent segment degeneration- (ASD-) free time from the initial surgery.

**Figure 4:** Representative images from the case of a 61-year-old female with L4 spondylolisthesis. (a) Postoperative lateral radiographs at 2 weeks and 5 years after surgery. Posterior slippage of the L3 vertebra and decrease in L3/4 disc space height were found. (b) Sagittal (upper panel) and axial (lower panel) MRI images at L3/4 disc level at 2 weeks and 5 years after surgery. Posterior protrusion of the L3/4 disc (white arrow) is present at 5 years postoperatively. The axial view shows a decrease in the dural sac cross-sectional area and thickening of connective tissue and ligaments around the facets at 5-year follow-up. (c) Preoperative CT axial view at the L3/4 facet joint shows overall joint space narrowing and a subchondral cyst (white arrow).

**Table 1:** Patients demographic data and surgical outcomes.

*N*	41	
Sex		
Male	18 (43.9%)	
Female	23 (56.1%)	
Mean age (yrs)	70.0 ± 7.2	
Diagnosis		
Degenerative spondylolisthesis	33 (80.5%)	
Grade 1	31	
Grade 2	2	
Spinal canal stenosis	8 (19.5%)	
Type of posterior fixation		
Indirect decompression (PPS)	41 (100%)	
Graft materials		
Autografts and bone graft substitutes	41 (100%)	
Number of fixation levels		
1 level	31 (75.6%)	
2 levels	10 (24.3%)	
Fixation vertebral levels (including duplicate)		
L3/4	15	
L4/5	36	
Combined with adjacent segment decompression	0	
Clinical surgical outcomes		
Preop. JOA score	14.8 ± 4.3	
Postop. JOA score (vs. preop.)	25.8 ± 2.5	(<0.001)
Radiographical surgical outcomes		
Preop. LL (degree)	41.2 ± 12.4	
Postop. LL (degree) (vs. preop.)	44.1 ± 13.4	(0.007)
Preop. PI-LL mismatch (degree)	9.1 ± 11.8	
Postop. PI-LL mismatch (degree) (vs. preop.)	6.2 ± 12.0	(0.007)
Preop. local lordosis (degree)	6.9 ± 7.2	
Postop. local lordosis (degree) (vs. preop.)	13.1 ± 5.2	(<0.001)
Preop. intervertebral height (mm)	8.6 ± 4.2	
Postop. intervertebral height (mm) (vs. preop.)	13.8 ± 4.7	(<0.001)
Radiographical parameters at cranial adjacent level		
Facet joint osteoarthritis		
1	6	
2	17	
3	15	
4	3	
Adjacent disc degeneration (Pfirrmann grading system)		
1	0	
2	1	
3	7	
4	24	
5	9	
Preop. dural sac cross-sectional area (mm^2^)	147.3 ± 36.4	
Postop. dural sac cross-sectional area (mm^2^) (vs. preop.)	140.3 ± 37.6	(0.005)
Facet joint violation, case	2 (4.9%)	

PPS: percutaneous pedicle screw; LL: lumbar lordosis; PI: pelvic incidence.

The article "Impact of Adjacent Facet Joint Osteoarthritis on Adjacent Segment Degeneration after Short-Segment Lateral Lumbar Interbody Fusion for Indirect Decompression: Minimum 5-Year Follow-Up" was published in 2022. Journal: Biomed Res Int.

**Table 2:** Five-year outcomes of the ASD+ and ASD- groups.

	ASD+ group	ASD- group	*P*
*N*	14	27	
Reoperation	2 (14.3%)	0	0.111
Clinical outcome			
Change of JOA score (vs. postop.)	−2.3 ± 3.4	−1.1 ± 3.2	0.266
Symptomatic	4 (28.6%)	6 (22.2%)	0.712
Radiographical outcomes			
Bony fusion	13 (92.9%)	23 (85.2%)	0.645
Radiographical parameters at cranial adjacent level			
Deterioration of disc degeneration (Pfirrmann grading system)	12 (85.7%)	6 (22.2%)	<0.001
Change of dural sac cross-sectional area (%) (vs. post op.)	−28.1 ± 25.3	−10.4 ± 22.4	0.027

ASD: adjacent segment degeneration; JOA: Japanese Orthopaedic Association.

**Table 3:** Analysis of risk factors of ASD, patient characteristics, and postoperative radiographical parameters.

	ASD+ group (*N* = 14)	ASD- group (*N* = 27)	*P*
Age, years	71.1 ± 7.6	69.4 ± 7.0	0.494
Sex (female)	7 (50.0%)	16 (59.3%)	0.742
Number of fixation levels (2 levels)	6 (42.9%)	4 (14.8%)	0.064
Facet violation with PPS	2 (14.3%)	0	0.111
Radiographical parameters			
Postop. PI (degree)	48.4 ± 11.4	51.3 ± 9.8	0.432
Postop. PT (degree)	21.4 ± 7.7	21.7 ± 8.8	0.908
Postop. SS (degree)	30.2 ± 6.8	32.8 ± 7.5	0.313
Postop. LL (degree)	43.1 ± 14.9	44.6 ± 12.8	0.754
Postop. PI-LL mismatch (degree)	5.3 ± 12.1	6.7 ± 12.1	0.732
Acquisition of local lordosis (degree)	6.9 ± 6.7	5.8 ± 6.4	0.637
Acquisition of intervertebral height (mm)	5.9 ± 2.6	4.8 ± 2.0	0.165
Radiographical parameters at cranial adjacent level			
Preop. facet joint osteoarthritis			0.008
Grade 1	0	6	
Grade 2	4	13	
Grade 3	9	6	
Grade 4	1	2	
Preop. adjacent disc degeneration (Pfirrmann grading system)			0.566
Grade 1	0	0	
Grade 2	1	1	
Grade 3	6	12	
Grade 4	7	12	
Grade 5	0	2	

ASD: adjacent segment degeneration; PPS: percutaneous pedicle screw; PI: pelvic incidence; PT: pelvic tilt; SS: sacral slope; LL: lumbar lordosis.

The article "Impact of Adjacent Facet Joint Osteoarthritis on Adjacent Segment Degeneration after Short-Segment Lateral Lumbar Interbody Fusion for Indirect Decompression: Minimum 5-Year Follow-Up" was published in 2022. Journal: Biomed Res Int.

## Data Availability

The observational data used to support the findings of this study are available from the corresponding author upon request.
